# The Effect of Age on IVF-ET Outcome in Infertile Patients with PCOS Based on Tiangui Theory in Chinese Medicine

**DOI:** 10.1155/2022/2977636

**Published:** 2022-08-22

**Authors:** Hui Chang, Jian Li, Qi Wu, Xin Fu, Mengyi Zhu, Hang Ge, Baichao Shi, Xiaoguang Shao, Yanhua Han

**Affiliations:** ^1^Department of Obstetrics and Gynecology, First Affiliated Hospital, Heilongjiang University of Chinese Medicine, Harbin 150040, China; ^2^Heilongjiang University of Chinese Medicine, Harbin 150040, China; ^3^Affiliated Hospital of Guizhou University of Traditional Chinese Medicine, Guiyang 550000, China; ^4^Shenzhen Lachesis Mhealth Co., Ltd., Shenzhen 51800, China; ^5^Dalian Municipal Women and Children's Medical Center, Dalian 116037, China

## Abstract

**Objective:**

Our aim was to investigate the effect of age on the outcome of IVF-ET and ICSI in infertile PCOS patients under the guidance of Tiangui theory in traditional Chinese medicine.

**Method:**

This was a retrospective analysis of 532 infertile women with PCOS and 1,392 women with infertility due to tubal factors as the controls. All of the participants were divided into different age groups-aged 20–28 years, 29–35 years, and ≥36 years-according to the stages of female reproductive development in Tiangui theory as described in the Canon of Internal Medicine-Treatise of Ancient Natural Truth. We explored the effect of age on controlled ovarian hyperstimulation (including the initial dosage and duration of Gn and the estradiol level on the day of human chorionic gonadotropin administration); the numbers of retrieved oocytes, 2PN zygotes, and embryos; and the rates of fertilization, clinical pregnancy, abortion, live birth, and OHSS incidence.

**Results:**

Compared to controls, the maximum follicular diameter and the numbers of follicles with d ≥ 20 mm, retrieved oocytes, and 2PN zygotes were greater in the PCOS group with age >28 years (*p* < 0.05). The abortion rate of PCOS patients with age ≤28 years was higher than that of the controls. All PCOS groups and the control group showed reduced numbers of retrieved oocytes and live births with age. The difference in age was not significant in the PCOS groups but was significant in the control group (*p* < 0.05), and the trend in the PCOS groups was more gradual.

**Conclusion:**

The fertility of all subjects decreased with age, but PCOS patients decreased more slowly than in controls at the same age, which verified the applicability of the guiding principles of Tiangui theory in the clinic.

## 1. Introduction

Polycystic ovary syndrome (PCOS) is a fairly common endocrine disorder in young reproductive-age women. PCOS is a multifactorial disorder and is characterized by a combination of clinical (anovulation and hyperandrogenism), biochemical (excessive androgen and luteinizing hormone concentrations), and ovarian (polycystic ovaries) features [1]. Infertility is the main reason for PCOS patients of reproductive age to seek medical treatment, and current treatment measures include drug ovulation induction, laparoscopic ovarian drilling, or acupuncture to achieve the goal of ovulation induction and natural conception. However, 20% of patients still need assisted reproductive technology in order to conceive. Recently, it has been shown that the incidence of adverse pregnancy outcomes after in vitro fertilization-embryo transfer (IVF-ET) and intracytoplasmic sperm injection-embryo transfer (ICSI-ET) increases with age. Both the number and quality of follicles decrease in an age-dependent manner, especially in women over 35 years. After 38 years of age, follicular atresia accelerates sharply along with a lower pregnancy rate, higher abortion rate, and lower delivery rate. It has also been reported that although the clinical pregnancy rate in PCOS patients over 38 years is lower than in healthy women, the numbers of retrieved oocytes do not show significant differences [2]. In addition, Tannus and Colleagues found that PCOS patients over 40 years of age had higher oocyte numbers and a higher cumulative live birth rate than in healthy women of the same age [3].

In traditional Chinese medicine, Tiangui theory seeks to describe the development and maintenance of reproduction and expounds upon, how reproductive function varies at different stages in humans. For females, the length of one stage is 7 years. The filling and exhaustion of Tiangui, which is derived from the kidney essence, is closely related to female fertility. It is said in the Canon of Internal Medicine-Treatise of Ancient Natural Truth (hereafter referred to as the Internal Classic) that “Girls of seven years have abundant kidney qi, they get their adult teeth, and they grow long hair; at the second seven Tiangui arrives, the conception vessel circulates smoothly, the thoroughfare vessel is abundant, menstruation occurs regularly, and pregnancy is possible….” With the age changing from the third seven to the seventh seven, female fertility changes along with Tiangui's growth and cessation [4]. Premature ovarian failure is characterized as “Tiangui disorder.”

Based on Tiangui theory, we performed a retrospective analysis to investigate the effect of age on ovarian function and IVF-ET outcomes in infertile PCOS patients.

In this paper, we retrospectively analyzed the differences in ovarian function and IVF-ET reproductive outcomes among infertile PCOS patients at different ages under the guidance of age-dependent female fertility according to Tiangui theory.

## 2. Research Data

### 2.1. Research Subjects

This was a retrospective analysis of data collected from October 2009 to October 2016 in Dalian Municipal Women and Children's Medical Center. A total of 532 infertile PCOS patients who had undergone their first IVF/ICSI-ET cycle were selected as the research subjects along with 1,392 patients, who underwent IVF/ICSI-ET due to tubal factors as the controls.

### 2.2. Diagnostic Criteria

The diagnostic criteria for infertility were those in the 8th edition of Obstetrics and Gynecology [5], and the diagnostic criteria for PCOS were the 2012 revision of the Rotterdam criteria [4].

### 2.3. Exclusion Criteria

IVF/ICSI patients were excluded if they reported endometriosis, hypothyroidism, hyperprolactinemia, congenital adrenocortical hyperplasia, chromosomal abnormalities, ovarian surgery history, or other diseases affecting fertility.

### 2.4. Grouping

According to Tiangui theory, patients were divided into three groups based on age and female reproductive stage: group A (aged 20–28 years, which is equivalent to the fourth seven in the Internal Classic), group B (aged 29–35 years, which is equivalent to between the fourth and fifth seven in the Internal Classic), and group C (aged ≥36 years, which is equivalent to the fifth seven in the Internal Classic).

All IVF/ICSI-ET patients involved in the study provided informed consent, and the study protocol was approved by the ethics committee of Dalian Municipal Women and Children's Medical Center and the ethics committee of the First Affiliated Hospital, Heilongjiang University of Chinese Medicine.

## 3. Materials and Methods

### 3.1. Pretreatment

All PCOS patients started taking oral Diane-35 at 1 tablet/day on the third day of menstruation before the treatment cycle and continued for 21 days.

### 3.2. Controlled Ovarian Hyperstimulation (COH)

All patients underwent the long standard protocol of COH. Pituitary down-regulation was achieved with gonadotropin-releasing hormone agonist (GnRH-a) administered on Day 5 to Day 7 after ovulation or on the 21st day of the menstrual cycle if using oral contraceptives. The dose of GnRH-a was 0.05 mg or 0.1 mg daily (according to the ovarian response) by subcutaneous injection. Serologic examination and transvaginal ultrasonography inspection were performed after 14 to 21 days of application of GnRH-a. Treatment with recombinant follicle-stimulating hormone (rFSH) (Gonal-F) to promote ovulation was initiated until the day of human chorionic gonadotropin (hCG) injection when the serum estradiol (E2) level, luteinizing hormone (LH), and vaginal ultrasonography evaluation met the criteria of down-regulation (E2 ＜ 5 pg/ml, LH ＜ 5 IU/L, endometrial thickness <4-5 mm, and nonfunctional cysts). The starting dose of gonadotropin (Gn) was 112.5–225 IU based on the patient's age, antral follicle count, basal E2 level, and body surface area.

### 3.3. Oocyte Retrieval, Semen Treatment, and Insemination

The follicular development was monitored by transvaginal ultrasonography and serologic examination on the 6th day after oocyte retrieval. Once 2-3 follicles reached the diameter of 18 mm by transvaginal ultrasonography, 5000–10000 IU hCG was added at night to induce follicular maturation, and transvaginal oocyte retrieval was performed 34–36 h after injection. The partner of the patient needed to ejaculate once 2–7 days before oocyte retrieval and sperm were obtained by masturbation on the day of oocyte retrieval. The semen was placed in an aseptic sperm retrieval cup and liquefied after 30 minutes of standing, and the sperm were capacitated after separation, washing, and culturing. At 2–4 h after oocyte retrieval, IVF or ICSI was performed and the fertilization status was observed after 16–18 h. Normal fertilization results in the presence of two pronuclei or two polar bodies in the cytoplasm. Embryo evaluation was based on the criteria of Peter [6].

### 3.4. Embryo Transplantation and Clinical Pregnancy Detection

On the third day after oocyte retrieval, high-quality embryos were selected for transplantation when the patient's endometrial thickness was up to 8 mm and were selected according to the patient's age, endometrial receptivity, and risk of ovarian overstimulation. The remaining embryos were cryopreserved by vitrification. Luteal phase support was provided by oral, intramuscular injection, or intravaginal progesterone. At 14 days after embryo transfer, biochemical pregnancy was determined by serum hCG concentration, and 30 days later the position and number of gestational sacs were determined by transvaginal ultrasonography. Biochemical pregnancy was defined by serum *β*-hCG concentration >10 IU/L and the absence of a gestational sac detected by transvaginal ultrasonography. Clinical pregnancy was defined as an ultrasound finding of the pregnancy sac (intrauterine or extrauterine) with a heartbeat.

### 3.5. Primary Measurements

#### 3.5.1. Serum Hormone Levels Measurement

The fasting blood sample of patients was instructed to be taken on the second or third day of a regular menstrual cycle or after progesterone withdrawal bleeding. The serum levels of E2, LH, FSH, testosterone, prolactone, and thyroid stimulating hormone were monitored by microparticle enzyme immunoassay. A fasting blood sample was taken to detect serum E2 on the day of oocyte retrieval.

#### 3.5.2. Clinical Indexes Calculation

The implantation rate was calculated as the number of patients with fetal heartbeat observed under B-ultrasound divided by the number of transplanted embryos.

The rate of clinical pregnancy was calculated as the sum of the number of patients with fetal heartbeat observed under B-ultrasound and the number of patients with *β*-HCG-positive serum divided by the total number of subjects.

The fertilization rate was calculated as the number of patients with fertilization (including the presence of clinical pregnancy or abortion) divided by the total number of subjects.

The clinical pregnancy rate was calculated as the number of patients with more than 28 weeks of pregnancy divided by the total number of subjects.

The abortion rate was calculated as the number of patients with abortions that occurred 28 weeks ago divided by the total number of subjects.

The live birth rate was calculated as the number of patients with ≥28 weeks of pregnancy divided by the total number of subjects.

The incidence rate of OHSS was calculated as the number of patients with OHSS divided by the total number of subjects.

## 4. Statistical Analyses

All statistical analyses were performed using SPSS version 19.0. All data are shown as the mean and standard deviation. The comparisons between groups used a one-way analysis of variance. The numerical data were compared using the chi-squared test, and rates were compared using Fisher's exact test. *p* < 0.05 was considered statistically significant. The clinical pregnancy rate, live birth rate, and OHSS data with positive primary outcomes were analyzed by logistic regression.

## 5. Results

### 5.1. Baseline Characteristics of PCOS Patients

As shown in Table 1, the PCOS group had a higher BMI, longer duration of infertility, a lower initial dose of Gn, shorter duration of Gn use, higher LH and LH/FSH, and lower FSH compared with the control group (*p* < 0.05). The PCOS group above the age of 35 years had higher initial doses of Gn and lower E2 levels compared with the other two PCOS groups (*p* < 0.05).

### 5.2. Ovulation Induction Outcomes in PCOS Patients

As shown in Table 2, the maximum follicular diameter, number of follicles with d ≥ 20 mm, number of retrieved oocytes, and number of 2PN zygotes in the PCOS group B and group C were significantly higher compared with the group b and group c (*p* < 0.05).

### 5.3. Pregnancy Outcomes and Neonatal Outcomes in PCOS Patients

The implantation rate, clinical pregnancy rate, presence of clinical pregnancy rate, and live birth rate in the PCOS group aged ≥36 years were significantly lower than in the other two PCOS groups. The rate of abortion in the PCOS group aged 20–28 years was higher than the controls, while the OHSS rate in the PCOS group aged ≥36 years was significantly higher than the controls, and the difference remained significant after adjusting for BMI, the initial dose of Gn, and the duration of Gn. The days of pregnancy in the PCOS group aged ≥36 years was less than the controls (Table 3).

### 5.4. Comparison of the Number of Retrieved Oocytes and Live Birth Rate in PCOS Patients of Different Ages

With increasing age, the number of retrieved oocytes and the live birth rate in the PCOS groups did not decrease significantly (*p* > 0.05), while these all showed significant declines in the control group (*p* < 0.05) (The slope of the number of retrieved oocytes: PCOS group vs. control group = –0.028 vs. −0.25; the slope of the live birth rate: PCOS group vs. control group = −0.014 vs. −0.023) (Figures 1 and 2).

## 6. Discussion

Tiangui is first seen in the Internal Classic, which states, “Girls of seven years have abundant kidney qi, they get their adult teeth and grow long hair; at the second seven Tiangui arrives, the conception vessel circulates smoothly, the thoroughfare vessel is abundant, menstruation occurs regularly, and pregnancy is possible.” Tiangui is thus, closely related to female fertility. As the woman ages through the third seven, fourth seven, fifth seven, sixth seven, and seventh seven, Tiangui grows to a peak and then decreases leading to the eventual failure of female fertility [4]. The theory of the kidney qi-Tiangui thoroughfare-conception vessels-uterus reproductive axis is well established. Kidney qi gradually grows until it becomes exuberant, which promotes the emergence of Tiangui, and together they play a central role in the physiology of the uterus, and thus female fertility declines along with deficiency of kidney qi and the exhaustion of Tiangui [7]. Because the qi-blood and yin-yang relationships in the reproductive axis are disturbed in Tiangui disorders because kidney deficiency is a root aspect of PCOS and turbid phlegm is a branch aspect, PCOS patients usually have oligomenorrhea, anovulation, blocked thoroughfare vessel and conception vessel, and phlegm congestion in the uterus, and they present the main manifestations of obesity, hirsutism, acne, and other metabolic disorders. Invigorating the kidney and resolving phlegm are the starting points of treatment [8, 9].

It is currently proposed that PCOS patients might have a wider reproductive window than healthy women. Minooee et al. observed that PCOS patients have significantly higher serum anti-Müllerian hormone (AMH) than normal ovulatory women and that they might have a 2-year longer reproductive lifespan when compared with their normal ovulatory counterparts [10]. In terms of reproductive outcomes, a retrospective cohort study explored the effect of age on the cumulative live birth rate after the first ovarian stimulation in IVF in PCOS patients and showed that declines in treatment outcomes were slower in PCOS patients compared to non-PCOS patients [11]. However, another study found that clinical pregnancy and live birth rates between PCOS patients and women with tubal factor infertility were similar, and the hypothesis that the reproductive window is extended in PCOS patients was not supported [12].

Age is one of the predictors of ovarian reserve function and is an independent factor affecting female fertility. As women age, the number of follicles decreases along with a decline in ovarian reserve function, and the incidence of infertility in women aged 40 is twice as high as in women aged 30–35 [5]. AMH is generally considered the best currently available measure of ovarian reserve in various clinical conditions. Low AMH levels represent low ovarian reserve, and it is common for AMH levels to gradually decline as a woman ages [13]. Researchers have compared AMH mRNA expression in cumulus and mural granulosa cells and measured the AMH level in follicular fluid of women aged 21–35 years and 40–45 years. The expression of small noncoding microRNA also differs in the follicular fluid between PCOS patients and normal healthy women, and age is one of the factors, that is, correlated with these changes [14]. The results showed that AMH was highly expressed and secreted from cumulus granulosa cells in women of advanced age [15]. Another study of AMH levels at different ages among women receiving IVF-ET or ICSI treatment found a statistically significant difference in AMH between groups aged 24–30 and 41–45 years. When it comes to pregnancy rates, significant differences were seen between groups aged under 30 and other groups, as well as between the groups aged 31–35 and 41–45 years [16]. It can thus be speculated from the studies above that the decline of ovarian function is more obvious in women over 40 years old.

An analysis of the follicular fluid of IVF patients at different ages found that with the increase in age the quality and quantity of oocytes tended to decline, while the level of reactive oxygen species gradually increased in follicles, and the follicular fluid microenvironment, which is closely related to the development of the oocyte, also changed [17]. Shi Li-hong et al. [18] found that the live birth rate and abortion rate of IVF patients over the age of 43 who underwent the long protocol of COH were reduced and increased, respectively, and they proposed that age was an independent factor affecting the pregnancy outcome of IVF-ET attempts. For women over 37 years old receiving IVF/ICSI-ET, the clinical pregnancy decreased and the spontaneous abortion rate increased with increasing age, especially for women over 44 years old. This is consistent with the traditional Chinese medicine notion that “At the fifth seven, the Yangming meridian starts to decline, her face begins to wither, and her hair begins to thin” and supports the theory of changes in female fertility at different ages. The fertility window of PCOS patients may extend to 40 years of age, but at ages, over 40 years old come declining ovarian reserve, the poor effect of ovulation-stimulating treatments, and a low pregnancy rate [19]. Despite serum AMH decreases over time in all of the women, the decrease in the PCOS patients was less pronounced than in controls, and this may suggest better preservation of the ovarian reserve and thus a prolonged reproductive life span [20]. A study showed that the live birth rate and cumulative live birth rate in PCOS patients aged 35–40 years were significantly higher than in the control group [11]. In another study, AMH levels in PCOS patients aged 20–30 and those aged 30–40 were not significantly different, but in non-PCOS patients AMH levels in the group aged 20–30 were significantly higher than those in the group aged 30–40 [21]. It has been reported that the threshold of AMH might be more accurate in predicting PCOS based on age stratification, which may account for the difference in age-related AMH levels between PCOS patients and healthy women [6]. Moreover, it has been shown that AMH levels gradually decrease with age, although the rate of AMH decline may not be the same for all women of reproductive age. There is also evidence that the ovarian pool is depleted in a more gradual manner in the ovaries of PCOS patients compared to healthy women [22].

In this study, the number of retrieved oocytes, 2PN zygotes, and embryos formed in the controls showed a significantly decreasing trend with increasing age, whereas there were no differences in the PCOS group with age but they were all higher than the control group (*p* < 0.05). The number of retrieved oocytes is an important indicator of ovarian function, suggesting that PCOS patients have a better ovarian reserve function according to the results of this study. Meanwhile, we found that the implantation success rate, conception rate, clinical pregnancy rate, ongoing pregnancy rate, and live birth rate both in the PCOS group and control group declined with age and were greater in the PCOS group compared to the control group but the differences were not statistically significant. A study indicated that the number of retrieved oocytes, the pregnancy rate, and the live birth rate in PCOS patients remained relatively stable but showed a significant decreasing trend in the control group [23]. This was consistent with our results (Figure 2), which indicated that the ovarian function in PCOS patients was better than that in healthy women of the same age.

In this study, the rate of abortion in the PCOS group aged 20–28 years was higher than that in the control group, while the OHSS incidence rate in the PCOS group aged ≥36 was higher than in the control group, and both remained significantly different after adjusting for BMI, the initial dose of Gn, and the duration of Gn. This indicated that the high abortion rate in PCOS patients before the age of 28 may be related to changes in the uterine and endocrine environment needed to maintain pregnancy, while the ovaries have a relatively good reserve and response over 35 years, resulting in the higher risk of OHSS occurrence. Hwang [2] found that the number of retrieved oocytes remained stable and that the conception rate, clinical pregnancy rate, and live birth rate declined in the PCOS group with age, but were superior to controls. The women with PCOS had a lower miscarriage rate than the controls, although it increased with age. This finding also supports our hypothesis that the decrease in fertility with age is slower in PCOS than in controls and suggests that ovarian reserve function was superior in PCOS compared with the control group at the same age.

Our study has several strengths. It is the first to evaluate IVF outcomes with Tiangui theory of TCM, which provides clinical evidence in support of Tiangui theory of TCM. We found that fertility in the women declined with age but the fertility in PCOS might be superior to that of the control group. Furthermore, it had a large sample size with a total of 532 infertile women with PCOS and 1924 women with tubal factor infertility who did not have PCOS, which has important significance for clinical guidance. A limitation of this study is that this was a retrospective analysis and some important indicators could not be collected, such as AMH, which is one of the most important factors for predicting ovarian reserve function, and thus these values were not fully tested in this paper.

## Figures and Tables

**Figure 1:** Age-related changes in the number of retrieved oocytes. The number of retrieved oocytes declined with age both in the two groups, while the number of retrieved oocytes in the PCOS group was significantly better than that in the control group.

**Figure 2:** Age-related changes in the live birth rate. The live birth rate declined with age both in the two groups, while the live birth rate in the PCOS group was significantly better than that in the control group, as the change in the number of retrieved oocytes.

**Table 1:** The baseline characteristics of PCOS patients.

	PCOS			Tubal factor		
	Group A age, 20–28	Group B age, 29–35	Group C age, ≥36	Group a age, 20–28	Group b age, 29–35	Group c age, ≥36
Subjects (*n*)	81	350	101	114	753	525
Age (years)	26.7 ± 1.4	32.0 ± 1.9	38.3 ± 2.1^#^	26.7 ± 1.5	32.4 ± 1.9	38.6 ± 2.3^#^
BMI (kg/m^2^)	23.9 ± 3.6^*∗*^	23.9 ± 3.4^*∗*^	24.6 ± 4.0^*∗*^	21.5 ± 3.0	22.6 ± 3.3	22.8 ± 2.9^#^
Duration of infertility (years)	3.3 ± 1.6^*∗*^	4.3 ± 2.6^*∗*^	6.3 ± 4.1^*∗*^^#^	2.7 ± 1.8	4.0 ± 2.8	5.6 ± 4.4^#^
Initial dose of Gn (IU)	159.5 ± 59.5^*∗*^	182.7 ± 64.9^*∗*^	212.4 ± 76.4^*∗*^^#^	196.4 ± 75.3	243.2 ± 68.5	276.9 ± 64.3^#^
Duration of Gn use (days)	9.3 ± 2.0^*∗*^	9.4 ± 2.7^*∗*^	10.7 ± 2.1^*∗*^	9.9 ± 1.7	10.2 ± 1.9	11.2 ± 2.3
LH (U/L)	6.6 ± 3.6^*∗*^	6.3 ± 4.1^*∗*^	6.3 ± 5.0^*∗*^	4.6 ± 2.4	4.3 ± 2.0	4.2 ± 1.8
FSH (U/L)	6.6 ± 2.3^*∗*^	6.7 ± 2.0^*∗*^	7.0 ± 2.0^*∗*^	7.3 ± 2.1	7.5 ± 2.2	9.5 ± 33.8^#^
LH/FSH	1.2 ± 1.6^*∗*^	0.95 ± 0.5^*∗*^	0.9 ± 0.7^*∗*^	0.7 ± 0.4	0.6 ± 0.3	0.6 ± 0.6^#^
E2 (pg/ml)	40.9 ± 26.2	36.9 ± 16.8	36.5 ± 15.2^*∗*^^#^	38.6 ± 21.7	40.6 ± 22.5	42.1 ± 22.2

^*∗*^ *p* < 0.05 compared with control at the same age. ^#^*p* < 0.05 compared within the PCOS group and control group.

**Table 2:** The comparison of ovulation induction outcomes in PCOS patients of different ages.

	PCOS			Tubal factor		
	Group A age, 20–28	Group B age, 29–35	Group C age, ≥36	Group a age, 20–28	Group b age, 29–35	Group c age, ≥36
Subjects (*n*)	81	350	101	114	753	525
E2 level on the day of hCG injection (pg/ml)	3487.9 ± 2038.1	3103.9 ± 1879.1	2472.5 ± 1686.6^*∗*^	3156.8 ± 2123.0	2945.3 ± 1851.7	2441.4 ± 1829.1^#^
Maximum follicular diameter (mm)	22.6 ± 1.8	22.5 ± 2.1^*∗*^	22.9 ± 1.5^*∗*^	22.5 ± 1.6	22.3 ± 1.7	21.8 ± 1.5^#^
Number of follicles with d ≥ 20 mm	3.6 ± 1.9	3.4 ± 1.7^*∗*^	3.7 ± 2.0^*∗*^	3.2 ± 1.6	2.9 ± 1.5	2.3 ± 1.4^#^
Number of retrieved oocytes	7.9 ± 3.7	8.3 ± 3.8^*∗*^	7.5 ± 3.3^*∗*^	8.4 ± 3.2	7.6 ± 3.4	4.8 ± 2.9^#^
Number of 2PN zygotes	6.8 ± 3.5	6.8 ± 3.2^*∗*^	6.2 ± 3.1^*∗*^	6.8 ± 2.8	6.1 ± 3.0	4.8 ± 2.9^#^
Number of embryos	5.5 ± 2.8	5.5 ± 2.8	5.1 ± 2.8^*∗*^	6.2 ± 2.9	5.3 ± 2.9	4.1 ± 2.5^#^

^*∗*^ *p* < 0.05 compared with control at the same age. ^#^*p* < 0.05 compared within the PCOS group and control group.

**Table 3:** The pregnancy outcomes and neonatal outcomes in PCOS patients.

	PCOS			Tubal factor		
	Group A age, 20–28	Group B age, 29–35	Group C age, ≥36	Group a age, 20–28	Group b age, 29–35	Group c age ≥36
Subjects (*n*)	81	350	101	114	753	525
Number of embryos transferred	166	779	269	248	2494	1369
Implantation rate (%)	74/166^*∗*^	252/779^*∗*^	58/269^*∗*^^#^	79/248	479/2494	227/1369^#^
Fertilization rate (%)	53/81	198/350	45/101^#^	62/114	390/753	198/525^#^
Clinical pregnancy rate (%)	45/81	175/350	38/101^#^	58/114	352/753	167/525^#^
Presence of clinical pregnancy rate (%)	41/81	153/173	29/101^#^	53/114	305/753	128/525^#^
Abortion rate (%)	16/53^*∗*^^a^	49/198	16/45	9/114	87/390	71/198^#^
Live birth rate (%)	37/81	149/350	29/101^#^	53/114	303/753	127/525^#^
Ectopic pregnancy rate (%)	2/81	7/350	2/101	3/114	10/753	7/525
OHSS incidence rate (%)	1/81	6/350	4/101^*∗*^^a^	1/114	11/753	3/525
Neonatal weight (g)	2909 ± 664.8	2958 ± 696.7	2881 ± 844.8	2948 ± 562.8	2990 ± 623.0	2931 ± 625.3
Duration of pregnancy (d)	262.7 ± 16.8	265.8 ± 16.0	261.7 ± 16.9^*∗*^	264.1 ± 13.0	265.5 ± 14.5	268.2 ± 16.3

^*∗*^ *p* < 0.05 compared with control at the same age. ^#^*p* < 0.05 compared within the PCOS group and control group. ^a^*p* < 0.05 compared with control at the same age after adjusting for BMI, the initial dose of Gn, and the duration of Gn.

## Data Availability

The data are available from the corresponding author upon request.
